# Dealing with false positive risk as an indicator of misperceived effectiveness of conservation interventions

**DOI:** 10.1371/journal.pone.0255784

**Published:** 2021-08-05

**Authors:** Igor Khorozyan

**Affiliations:** Department of Conservation Biology, Georg-August-Universität, Göttingen, Germany; Qinghai University, CHINA

## Abstract

As human pressures on the environment continue to spread and intensify, effective conservation interventions are direly needed to prevent threats, reduce conflicts, and recover populations and landscapes in a liaison between science and conservation. It is practically important to discriminate between true and false (or misperceived) effectiveness of interventions as false perceptions may shape a wrong conservation agenda and lead to inappropriate decisions and management actions. This study used the false positive risk (FPR) to estimate the rates of misperceived effectiveness of electric fences (overstated if reported as effective but actually ineffective based on FPR; understated otherwise), explain their causes and propose recommendations on how to improve the representation of true effectiveness. Electric fences are widely applied to reduce damage to fenced assets, such as livestock and beehives, or increase survival of fenced populations. The analysis of 109 cases from 50 publications has shown that the effectiveness of electric fences was overstated in at least one-third of cases, from 31.8% at FPR = 0.2 (20% risk) to 51.1% at FPR = 0.05 (5% risk, true effectiveness). In contrast, understatement reduced from 23.8% to 9.5% at these thresholds of FPR. This means that truly effective applications of electric fences were only 48.9% of all cases reported as effective, but truly ineffective cases were 90.5%, implying that the effectiveness of electric fences was heavily overstated. The main reasons of this bias were the lack of statistical testing or improper reporting of test results (63.3% of cases) and interpretation of marginally significant results (p < 0.05, p < 0.1 and p around 0.05) as indicators of effectiveness (10.1%). In conclusion, FPR is an important tool for estimating true effectiveness of conservation interventions and its application is highly recommended to disentangle true and false effectiveness for planning appropriate conservation actions. Researchers are encouraged to calculate FPR, publish its constituent statistics (especially treatment and control sample sizes) and explicitly provide test results with p values. It is suggested to call the effectiveness “true” if FPR < 0.05, “suggestive” if 0.05 ≤ FPR < 0.2 and “false” if FPR ≥ 0.2.

## Introduction

Large-scale and ever accelerating pressures of human activities on the environment urge for the implementation of practical, socially acceptable and effective interventions in biodiversity conservation [1,2]. The overall goal of such interventions is to prevent anthropogenic threats, reduce conflicts with wildlife and between stakeholders, and to recover local populations, landscapes and ecological functions [3–5]. The examples of conservation interventions are many, from locally applied electric fences to reduce damage or boost survival of fenced populations [6–8] to globally important protected areas aimed at curbing biodiversity loss [9]. Reduction-aimed interventions strive to reduce negative outcomes, such as poaching or damage by wildlife, and addition-aimed interventions are used to increase positive outcomes, such as species survival or richness [10]. Selection of most effective interventions and their wide applications are pivotal to build bridges between science and conservation and to foster good practices [11].

One of the most important, but rarely asked, questions faced during intervention applications is how to disentangle true and false (or misperceived) effectiveness from the scientific estimates of intervention effectiveness. This issue is practically important as false perceptions may shape a wrong conservation agenda and lead to inappropriate decisions and management [12,13]. For instance, translocation of conflict-causing predators to remote areas has been perceived and widely used as an effective intervention even though in practice it can be costly, cause high mortality of captured animals, or trigger more conflict [14,15]. As another example, underestimation of adverse impacts of invasive species on native biodiversity may hinder ecological research, bias knowledge and applications, and delay restoration actions [16,17]. All this tends to create complacency and demotivates practitioners and managers to find alternative, more efficient solutions. Misperceived effectiveness can be overstated when an intervention is reported as effective but statistically it is not, or understated when the scenario is opposite. This kind of uncertainty is incorporated in statistical estimates [18,19], but is often ignored by conservation scientists yet the concept of false positives and negatives is rather common in species identification, genetics, distribution and monitoring [20–22]. False positive risk provides a clue to the understanding of which intervention applications are truly effective and which are ineffective.

Effectiveness of interventions is usually measured by means of null hypothesis significance testing which, in its turn, relies on p values. The most commonly used threshold is p = 0.05, allowing the researchers to interpret sample variables with p < 0.05 as significantly different and those with p ≥ 0.05 as having no evidence of difference between specified treatment (with intervention) and control (without intervention) samples. In the meantime, the value of 0.05 implies that some differences claimed to be true (i.e. having p < 0.05) are actually false as they occur by chance [23]. The probability of such misidentified cases is called the false positive risk (FPR), which at p = 0.05 is equal to 0.26–0.29 meaning that 26–29% of cases are false positives [24,25]. The (mis)use of p values and ignorance of FPR is still widespread in ecology, in contrast to such disciplines as medicine, psychology and economics which began to doubt p values and search for substitutes much earlier [19,26]. Admitting that the use of p values is a deeply rooted practice that cannot be easily changed, some scientists suggest to raise a bar of statistical significance from p = 0.05 to p = 0.005 [19], measure FPR directly and avoid the notion “statistical significance” at all [25,27,28]. From a conservative standpoint, this means that only intervention applications having low FPR, such as 0.05 (5% risk) and lower, can be considered as truly effective.

Statistical considerations, such as those described above, are based on simulations with fictitious, usually normally distributed, data [25]. How perceived effectiveness reported by researchers fits effectiveness statistically proven by FPR in real studies is poorly understood. It can be assumed that the share of cases with misperceived effectiveness should be high due to unreported FPR. Even worse than ignorance of FPR is the fact (see the Results and Discussion of this study) that many studies report the effectiveness of a given intervention for granted and either conduct no statistical tests or provide insufficient data for independent verification. This poses a serious threat to planned or ongoing biodiversity conservation actions by providing information which in many cases can be wrong. Therefore, it is essential to explore real-world data on commonly used interventions so that to compare perceived vs. FPR-proven effectiveness across large samples of studies and make conclusions of broad relevance.

The aim of this study was to determine the extent to which the effectiveness of conservation interventions is misperceived, namely overstated and understated, in real applications. Electric fences were used as an example of interventions because they have been widely used since the 1930s [29], well published in the literature, and thus can provide broad implications over large scales [30]. The focus of the study was on estimating the rates of effectiveness misperceptions, explaining their causes, and offering recommendations on how to recognize them and improve the representation of true effectiveness of conservation interventions.

## Results

The search yielded 235 publications, of which 185 complied with the exclusion criteria and were left out. I used the remaining 50 publications which provided information on 109 cases (S1 Data). Out of these 109 cases, 88 were reported in the literature as effective and 21 as ineffective (Table 1). Sixty-nine cases (63.3%) did not use tests or show their results in distinguishing between effective and ineffective fencing. Eleven cases (10.1%) were reported to be effective even though their results were provided at unknown levels of p < 0.05 and statistically marginal levels of p < 0.1 and p around 0.05.

**Table 1:** Distribution of the numbers of reported and statistically proven effective and ineffective cases of electric fence applications under the thresholds of (a) FPR = 0.2, (b) FPR = 0.1 and (c) FPR = 0.05.

**a. Threshold FPR = 0.2**		**Statistically proven cases**		**Total**
		**Effective (FPR < 0.2)**	**Ineffective (FPR ≥ 0.2)**	
**Reported cases**	**Effective**	60	28	88
	**Ineffective**	5	16	21
**Total**		65	44	109
**b. Threshold FPR = 0.1**		**Effective (FPR < 0.1)**	**Ineffective (FPR ≥ 0.1)**	
**Reported cases**	**Effective**	52	36	88
	**Ineffective**	3	18	21
**Total**		55	54	109
**c. Threshold FPR = 0.05**		**Effective (FPR < 0.05)**	**Ineffective (FPR ≥ 0.05)**	
**Reported cases**	**Effective**	43	45	88
	**Ineffective**	2	19	21
**Total**		45	64	109

Electric fences were reported to be more effective in reduction-aimed cases and less effective in addition-aimed cases (χ^2^ = 9.751, df = 1, p = 0.002), but the effect size of this relationship was low to medium (Cramer’s V = 0.299). In contrast, FPR did not differ between reduction-aimed and addition-aimed cases (Kruskal-Wallis H = 1.052, df = 1, p = 0.305), nor did it differ between species (H = 7.871, df = 6, p = 0.248). FPR varied between studies (H = 75.206, df = 49, p = 0.009) and it was significantly lower in reported effective cases than in reported ineffective ones (H = 23.894, df = 1, p < 0.001).

The median ± SE of FPR was 0.05 ± 0.02 for reported effective cases and 0.58 ± 0.05 for reported ineffective cases (Fig 1). Despite this, in 28 out of 88 effective cases (31.8%) FPR was 0.22–0.54 indicating the rate of overstated perceived effectiveness at threshold FPR = 0.2 to be 31.8% (Table 1). Five out of 21 ineffective cases (23.8%) had FPR = 0.0001–0.18 so the rate of understated perceived effectiveness at threshold FPR = 0.2 was 23.8% (Table 1). The error rate at FPR = 0.2 was 30.3% over 109 cases (Table 1). At thresholds FPR = 0.1 and FPR = 0.05, the rate of overstated perceived effectiveness increased to 40.9% (36/88) and 51.1% (45/88), the rate of understated perceived effectiveness decreased to 14.3% (3/21) and 9.5% (2/21), and the error rate increased to 35.8% and 43.1%, respectively (Table 1; Fig 2).

**Fig 1:** Distribution of false positive risk (FPR) in reported effective and ineffective cases of electric fence applications. The shaded area demarcates the area above the threshold of FPR = 0.2 where cases are statistically proven to be ineffective. The ranges of FPR for overstated (reported as effective, but actually not as FPR ≥ 0.2) and understated (reported as ineffective, but actually effective as FPR < 0.2) perceived effectiveness are shown. The lower is the threshold FPR (0.1 and 0.05 in this study), the wider is the range of overstated perceived effectiveness and the narrower is the range of understated perceived effectiveness.

**Fig 2:** Changes in rates of overstated perceived effectiveness, understated perceived effectiveness and error (misclassification) depending on threshold false positive risk (FPR) values.

## Discussion

This study has demonstrated that the effectiveness of electric fences was overstated (falsely claimed as effective) in at least one-third of cases described in the scientific literature (Table 1; Fig 1), regardless of the species and purposes of electric fencing. When FPR was set at 20% risk corresponding to the significance level p = 0.05 down to the desired 5% level of risk, the rates of overstated effectiveness increased from 32% to 51% and the rates of understated (falsely claimed as ineffective) effectiveness dropped from nearly 24% to almost 10% (Fig 2). This means that truly effective applications of electric fences made only 49% of all cases that reported this intervention as effective, but the share of truly ineffective cases in all cases reported as ineffective was much higher, 90%. For this reason, misperception of effectiveness was heavily biased towards its overstatement while most of ineffective cases were actually so. Another type of misinterpretation was that reduction-aimed applications of electric fences were perceived to be more effective than addition-aimed applications, but FPR-based statistical evidence did not find support for this difference.

Now the question arises why the effectiveness of so many electric fence applications is overstated. The most obvious reason was the lack of rigor in measurements and their reporting as in over 63% of cases no tests were used or their results were provided incompletely. Interestingly, lack or insufficient representation of effectiveness testing was found not only in old publications as it might be expected, but also in recent studies [6,31,32]. Another issue is that in 10% of cases the authors interpreted marginally significant results at p < 0.05, p < 0.1 and p around 0.05 as effective [7,33–37], but FPR has proved that none of cases at p < 0.1 and near 0.05, and only a half of cases at p < 0.05 were robust enough.

To be confident that the effectiveness of interventions is true, researchers are encouraged to calculate and publish FPR and also to provide (optimally, in tabular form) basic statistics of the treatment and control samples for independent verification and better understanding of study results. These basic statistics include the means, standard deviations, sample sizes, and effect sizes such as Cohen’s d. Statistical errors and 95% confidence intervals can be published as an alternative to standard deviations or provided in addition to them [24,26]. Of particular importance is to publish treatment and control sample sizes, especially for small samples [18], to avoid ambiguities and misunderstanding. Explicit representation of tests and their results is essential, with p values to be reported as exact numbers and never as p < 0.05 or p > 0.05.

The use of p values is ubiquitous and the replacement of this practice is not realistic, at least in effectiveness studies where null hypothesis significance testing reliant on p values is still the main approach. Even though the use of effect size metrics like relative risk, odds ratio, magnitude of change and Hedge’s d becomes more common to estimate effectiveness [10], testing can be useful to provide additional support for conclusions. Application of information-theoretic approaches using Akaike Information Criterion (AIC) and similar criteria is the most popular alternative to the use of p values in ecology, and the interest in Bayesian methods is increasing [26,28,38]. As the use of p values is expected to be practised for long, I concur with [28] that the best option is to supplement p values with more statistical data as mentioned above. It is suitable to measure FPR at prior probability of real effect p(H1) = 0.5 or to measure true effectiveness at FPR = 0.05, as it was done in this study. Similar to recommendations by [19], it is practical and informative to call the effectiveness “true” if FPR < 0.05, “suggestive” if 0.05 ≤ FPR < 0.2 and “false” if FPR ≥ 0.2.

This study has shown that FPR of the estimates of the effectiveness of electric fences significantly differed between studies, thus stressing the role of local contexts in successes or failures of this intervention. The effectiveness of electric fences depends on their maintenance to keep electric charge strong and constant, fence design, size of the fenced area, landscape topography, soil humidity and conductivity, and the coverage of the fence to prevent animals jumping over or sneaking under [33,34,37,39–41]. However, the pivotal role of these practical factors should not downplay the importance of statistical testing; instead, these two facets should go hand in hand to provide strong evidence for conservation.

Previous meta-analyses of the effectiveness of anti-predator interventions have shown that electric fences are among the most effective approaches to limit predator movements and reduce damage to fenced assets, such as livestock or beehives [8,11,42–47]. Yet, the present study demonstrated that a significant part of electric fence applications holds insufficient statistical evidence to support the effectiveness of this intervention. These conclusions are not contradictory because the mentioned meta-analyses are focused on mammalian predators, whereas this study included applications of electric fences to the species from crayfish (*Orconectes rusticus* and *O*. *meeki*) [48,49] and honey bees (*Apis mellifera*) [32] to African elephants (*Loxodonta africana*) [39], which in some cases were indeed variable and unreliable. Further, due to limitations imposed on specific statistical data required to calculate FPR, only eight cases of electric fencing were included in meta-analyses and this study (large predators [40,41,50,51], mesopredators [52–54], predators in general [55]).

In conclusion, this study has demonstrated that FPR is an important statistical tool of estimating true effectiveness of conservation interventions and its application is highly recommended to separate the cases of true and false effectiveness for planning appropriate conservation actions.

## Materials and methods

### Data sources

A comprehensive approach was used to extract the literature on the effectiveness of electric fences in wildlife applications. At the beginning, I selected relevant publications from the meta-analyses of the effectiveness of anti-predator interventions [8,11,42–47], as well as from the synopsis of effectiveness studies related to mammals [5]. Then I searched through Web of Science (www.webofknowledge.com, 1945–2020), BioOne (www.bioone.org, 1965–2020) and IUCN/SSC Cat Specialist Group Digital Library (www.catsg.org, 1950–2020) using the words “electric fenc*”. I checked all issues of Conservation Evidence (www.conservationevidence.com, 2004–2020), Carnivore Damage Prevention News (www.lcie.org and www.medwolf.eu, 2000–2005 and 2014–2020), Ursus (www.bearbiology.org and www.bioone.org, 1968–2020) and publications from the “Electric fences” section of the IUCN/SSC Human-Wildlife Conflict Task Force Library (www.hwctf.org). I scanned the ENCOSH (Enhancing Co-existence Through Sharing) online platform (www.encosh.org) and used snowball sampling of references from the literature. I ended the search on 24 July, 2020.

A study of electrified fladry, which is the rope with red flags serving as a deterrent against wolves (*Canis lupus*), was also considered because the effect of electric shocks lasts much longer than that of proper fladry [56]. I excluded the studies which did not contain required data or had insufficient data (see Data collection below), contained only one treatment or control replicate (so no standard deviation could be calculated), or applied regression analysis without control groups.

### Data collection

A dataset consisting of individual study cases was prepared for the analysis. Each case represented an electric fence application to protect a particular site from a particular species. The species were considered in general or as an individual species depending on how they were described by the authors. Whenever sufficient information was available on different fence designs, species or sites in a publication, they were considered as separate cases. Therefore, one publication could include several cases.

The following statistical parameters were collected for each case from publications, or calculated from the data therein: arithmetic means of treatment (${\bar{x}}_{t}$) and control (${\bar{x}}_{c}$) samples, sizes of treatment (N_t_) and control (N_c_) samples, and standard deviations of treatment (SD_t_) and control (SD_c_) samples. The samples with fence applications were considered as treatment samples, otherwise they served as control samples. If SD was not reported, it was calculated from the standard error SE as SD = SE ×√N or from the 95% confidence interval = $\bar{x}$ ± 1.96 × SE, taking the average SE from asymmetrical confidence intervals created by bootstrapping [57,58]. When $\bar{x}$ and SE were provided on graphs and not in the text, they were obtained using the Adobe Acrobat v. 9 Pro measuring tool. Effect size was calculated as Cohen’s d [28,59]:

$$Cohen's\;d=\frac{{\bar{x}}_{t}-{\bar{x}}_{c}}{\sqrt{\frac{(N_{t}-1)\times SD_{t}^{2}+(N_{c}-1)\times SD_{c}^{2}}{N_{t}+N_{c}-2}}}$$ (1)

where symbols are explained above. Negative values of Cohen’s d mean a decrease of the outcome of the treatment vs. control sample, zero means no effect, and positive values of Cohen’s d mean an increase of the outcome of the treatment sample [59,60]. For example, if the purpose of electric fences is to reduce livestock kills by predators or to increase the survival of bird nests, then these fences would be effective with negative Cohen’s d for livestock kills and with positive Cohen’s d for nest survival.

FPR was calculated for each case with the inputs of observed p value, prior probability of real effect p(H1), N_t_, N_c_ and Cohen’s d in FPR web calculator v. 1.7 (http://fpr-calc.ucl.ac.uk/, [61]). The statistical background of FPR calculation is provided in details in [25,27,28]. Observed p values were calculated through paired and independent t tests of treatment and control samples, depending on original study designs, with the inputs of $\bar{x}$, N, SD or paired samples in GraphPad QuickCalcs web calculator (www.graphpad.com). The “p-equals” and “p-less-than” options of FPR calculation were used for exact p values and p < 0.0001, respectively. Prior probability of real effect means the probability of the alternative hypothesis H1 (effectiveness of electric fences is statistically different in treatment vs. control) before the experiment is done. As the effectiveness of electric fences was not *a priori* known, p(H1) was set conservatively at 0.5, implying that the odds of electric fences to be effective or ineffective were 50:50 before these fences were experimentally tested [27,28]. The prior probability p(H1) = 0.5 produces the minimum estimate of FPR and the maximum of FPR = 1 is attained when p(H1) = 0 [25,28].

### Data analysis

The distribution of FPR across the studies, species, reported effectiveness of fencing and purpose of fencing was checked by Kruskal-Wallis test in IBM SPSS 26.0. This test was applied because FPR data were non-normal (Shapiro-Wilk statistic = 0.827, n = 109, p < 0.001). The species from which study sites were protected were categorized as aquatic species (fish and crayfish), birds (fish-eating), large predators, mesopredators (from martens to coyotes), small herbivores (hares and rabbits), ungulates, and others (mostly unspecified species). Reported effectiveness of fencing (effective or ineffective) and the purpose of electric fencing (reduction-aimed or addition-aimed, see Introduction) was recorded as the authors described them. It was recorded whether the division into effective and ineffective cases was supported by statistical tests or reported based on visual comparisons of treatment and control samples.

The graphical representation of FPR in reported effectiveness of fencing was provided by means of box plots. Chi-square (χ^2^) test in IBM SPSS 26.0 was used to check how the reported effectiveness of fencing was related to its purpose. Cramer’s V measured the effect size to vary from 0 (no association between effectiveness and purpose) to 1 (perfect association) [62].

A 2×2 contingency table was constructed to indicate how the numbers of reported effective and ineffective cases overlapped with the numbers of cases which were statistically proven by FPR to be effective and ineffective. Three thresholds were used to split the cases: (1) FPR < 0.2 as effective and FPR ≥ 0.2 as ineffective; (2) FPR < 0.1 as effective and FPR ≥ 0.1 as ineffective; and (3) FPR < 0.05 as effective and FPR ≥ 0.05 as ineffective. The threshold FPR = 0.20 corresponded to the threshold significance level of p = 0.05 (S1 Data) and FPR = 0.05 was the desired minimum level of risk (5%) when the effectiveness was true. The rate of overstated perceived effectiveness was quantified as a percentage of the number of false positive cases (N_10_), which reported electric fences to be effective but they were statistically ineffective as their FPR was ≥ threshold, to all reported effective cases. In opposite, the rate of understated perceived effectiveness was a percentage of the number of false negative cases (N_01_) reported as ineffective, but statistically effective with FPR < threshold, to all reported ineffective cases. In the statistical literature, the rate of overstated perceived effectiveness is denoted as the false discovery rate and the rate of understated perceived effectiveness is the false omission rate [63]. The error, or misclassification, rate was a percentage of the sum (N_10_ + N_01_) to the total number of cases in the study [63].

## Supporting information

S1 Data Raw data used in this study. (XLS)
